# A Post-training Quantization Method for the Design of Fixed-Point-Based FPGA/ASIC Hardware Accelerators for LSTM/GRU Algorithms

**DOI:** 10.1155/2022/9485933

**Published:** 2022-05-11

**Authors:** Emilio Rapuano, Tommaso Pacini, Luca Fanucci

**Affiliations:** Department of Information Engineering, University of Pisa, Pisa 56122, Italy

## Abstract

Recurrent Neural Networks (RNNs) have become important tools for tasks such as speech recognition, text generation, or natural language processing. However, their inference may involve up to billions of operations and their large number of parameters leads to large storage size and runtime memory usage. These reasons impede the adoption of these models in real-time, on-the-edge applications. Field-Programmable Gate Arrays (FPGAs) and Application-Specific Integrated Circuits (ASICs) have emerged as promising solutions for the hardware acceleration of these algorithms, thanks to their degree of customization of compute data paths and memory subsystems, which makes them take the maximum advantage from compression techniques for what concerns area, timing, and power consumption. In contrast to the extensive study in compression and quantization for plain feed forward neural networks in the literature, little attention has been paid to reducing the computational resource requirements of RNNs. This work proposes a new effective methodology for the post-training quantization of RNNs. In particular, we focus on the quantization of Long Short-Term Memory (LSTM) RNNs and Gated Recurrent Unit (GRU) RNNs. The proposed quantization strategy is meant to be a detailed guideline toward the design of custom hardware accelerators for LSTM/GRU-based algorithms to be implemented on FPGA or ASIC devices using fixed-point arithmetic only. We applied our methods to LSTM/GRU models pretrained on the IMDb sentiment classification dataset and Penn TreeBank language modelling dataset, thus comparing each quantized model to its floating-point counterpart. The results show the possibility to achieve up to 90% memory footprint reduction in both cases, obtaining less than 1% loss in accuracy and even a slight improvement in the Perplexity per word metric, respectively. The results are presented showing the various trade-offs between memory footprint reduction and accuracy changes, demonstrating the benefits of the proposed methodology even in comparison with other works from the literature.

## 1. Introduction

Deep Neural Networks (DNNs) are nowadays very popular tools for the resolution of any kind of task, ranging from finance and medicine to music, gaming, and various other domains. However, inference of a DNN may involve up to billions of operations and their high number of parameters leads to large storage size and runtime memory usage [1]. For this reason, a particular attention is given to the hardware acceleration of these models, especially when memory and power budgets are limited by the application constraints. This is the case of real-time, on-the-edge applications [2], where data elaboration is performed as close as possible to the sensors in order to guarantee benefits in terms of latency and bandwidth [3]. Modern solutions mostly use embedded Graphics Processing Units (GPUs), Field-Programmable Gate Arrays (FPGAs), and Application-Specific Integrated Circuits (ASICs) for the design of DNN hardware accelerators, choosing in dependence of several trade-offs concerning cost, performance, and flexibility [4, 5].

GPUs can handle very computationally expensive models in a flexible way, with the drawback of a reduced degree of customization which can lead to excessive power consumption, incompatibly with most on-the-edge applications [6, 7]. On the other hand, ASICs and FPGAs give the possibility to create specialized hardware that can be designed to minimize power consumption and area footprint while trying to keep a high throughput [8, 9]. In particular, FPGAs have emerged as a promising solution for hardware acceleration as they provide a good trade-off between flexibility and performance [10–12]. The main disadvantage of FPGA solutions consists in their limited hardware resources, making the hardware acceleration of complex DNN algorithms more challenging [11]. To alleviate DNNs storage and computation requirements, thus becomes an essential step to fit the limited resources of FPGA devices and to reduce the area footprint for a more efficient ASIC-based accelerator. With this purpose, many methods have been proposed from both hardware and software perspective [1]: techniques such as quantization and pruning are commonly applied to Neural Network models to reduce their complexity before hardware implementation. In contrast to the extensive study in compression and quantization for plain feed forward neural networks (such as Convolutional Neural Networks), little attention has been paid to reducing the computational resource requirements of Recurrent Neural Networks (RNNs) [1, 13, 14]. The latter have subtle and delicately designed structure, which makes their quantization more complex and needing for more careful considerations with respect to other DNN models. This work proposes a detailed description of a new effective methodology for the post-training quantization of RNNs. In particular, we focus on the quantization of Long Short-Term Memory (LSTM) RNNs [15] and Gated Recurrent Unit (GRU) RNNs [16], known in the literature as two of the most accurate models for tasks such as speech recognition [17], text generation [18], machine translation [19], natural language processing (NLP) [20], and movie frames generation [21, 22]. The proposed quantization strategy is meant to be a first step toward the design of custom hardware accelerators for LSTM/GRU-based algorithm to be implemented on FPGA or ASIC devices. With this purpose in mind, the results are presented showing the various trade-offs between model complexity reduction and model accuracy changes. The metric used to quantify model complexity is the estimated memory footprint needed for the hardware implementation of aLSTM/GRU accelerator after quantization. In summary, the main contributions of this work include the following:

- Detailed description of a new quantization method for LSTM/GRU RNNs which is friendly toward the energy/resource-efficient hardware acceleration of these models on ASICs or FPGAs
- Software implementation of LSTM/GRU quantized layers, compliant with the Python Tensorflow 2 framework [23].
- Evaluation of LSTM/GRU-based models' performance after quantization using the IMDb sentiment classification task and the Penn TreeBank (PTB) language modelling task

The paper is organized as follows: Section 2 gives an overview of the state of the art concerning LSTM/GRU models and the quantization techniques developed for them in the literature.  Section 3 describes in detail the proposed quantization strategy.  Section 4 discusses the results obtained with LSTM/GRU-based models pretrained on the IMDb sentiment classification dataset and on the PTB language modelling dataset.  Section 5 shows a comparison between the proposed method and other quantization algorithms taken from the literature. Finally, Section 6 draws the conclusions of this work.

## 2. Background

The traditional plain feed forward neural network approaches can only handle a fixed-size vector as input (e.g., an image or video frame) and produce a fixed-size vector as output (e.g., probabilities of different classes) through a fixed number of computational steps (e.g., the number of layers in the model) [24]. RNNs, instead, employ feedback paths inside that make them suitable for processing input data whose dimension is not fixed [24]. This characteristic makes them able to process sequences of vectors over time and keep “memory” of the results from previous timesteps, so that each new output will be produced with past information combined with the new coming input.

Among many types of RNNs [25, 26], two of the most used are LSTM [15] and GRU [16]. In particular, LSTM networks were designed to solve the gradient vanishing problem that makes standard Vanilla RNNs dependent from the length of the input sequence. On the other hand, GRU has become more and more popular, thanks to its lower computation cost and complexity. This work focuses on the quantization methods for these two kinds of RNN, chosen for their popularity within the literature so that we can make fair comparison. The LSTM and GRU functional schemes are depicted in Figures 1 and 2.

Pale yellow blocks constitute the so-called gates, divided into two categories depending on the activation function applied: tanh or sigmoid (indicated with the symbol *σ*). Pale red blocks are associated to pointwise operations. The gate mechanism makes these kinds of RNN a good option to deal with the vanishing gradient problem, since they can model long-term dependencies in the data. For what concerns the LSTM cell (Figure 1), the functionality of each gate can be summarized as follows:

- Forget gate: decides what information will be deleted from the cell state *c*_*t*−1_
- Input gate: decides which values of the input sequence (i.e., concatenation of current input *x*_*t*_ and previous output *h*_*t*−1_) will contribute to the state update
- Cell gate: creates a vector of new candidate values (*c*_*t*_′) that could be added to the state
- Output gate: decides the output of the cell *h*_*t*_ by combining information from the updated state *c*_*t*_ and current input sequence (*x*_*t*_, *h*_*t*−1_)

The four gates signals will be, respectively, referred with subscripts *f*, *i*, *c*, *o*. The following equations describe the mathematical behaviour of the LSTM cell [15].

(1) $$\begin{array}{c} \left\{\begin{array}{c} i_{t}=\sigma \left(x_{t}\cdot U_{i}+h_{t-1}\cdot W_{i}+b_{i}\right),\\ f_{t}=\sigma \left(x_{t}\cdot U_{f}+h_{t-1}\cdot W_{f}+b_{f}\right),\\ o_{t}=\sigma \left(x_{t}\cdot U_{o}+h_{t-1}\cdot W_{o}+b_{o}\right),\\ c_{t}^{\prime }=\tanh\left(x_{t}\cdot U_{c}+h_{t-1}\cdot W_{c}+b_{c}\right),\\ c_{t}=\sigma \left(f_{t}*c_{t-1}+i_{t}*c_{t}^{\prime }\right),\\ h_{t}=\tanh\left(c_{t}\right)*o_{t}. \end{array}\right. \end{array}$$

Each gate has its own weights matrices (*U* and *W*) and bias (*b*). *U* and *W* are, respectively, multiplied (through matrix-vector scalar product) with the current input vector *x*_*t*_ and with the cell output from previous timestep *h*_*t*−1_. The + and ∗ symbols are intended as pointwise sum and product operations, respectively.

On the other hand, the GRU model (Figure 2) is a significantly lighter RNN approach, with fewer network parameters since only three gates are used:

- Reset gate: decides the amount of past information (*h*_*t*−1_) to forget
- Update gate: decides what information to discard and what new information to add (acting similar to the forget and input gate of an LSTM)
- Output gate: decides the output of the cell *h*_*t*_

Keeping the same convention for symbols, but with gates subscripts being *r* (reset), *z* (update), *h* (output), the equations describing the GRU cell are the following [16]:

(2) $$\begin{array}{c} \left\{\begin{array}{c} z_{t}=\sigma \left(x_{t}\cdot U_{z}+h_{t-1}\cdot W_{z}+b_{z}\right),\\ r_{t}=\sigma \left(x_{t}\cdot U_{r}+h_{t-1}\cdot W_{r}+b_{r}\right),\\ h_{t}^{\prime }=\tanh\left[\left(x_{t}\cdot U_{h}\right.+\left(r_{t}*h_{t-1}\right)\cdot W_{h}+b_{h}\right],\\ h_{t}=\left[\left(1-z_{t}\right)*h_{t}^{\prime }\right]+\left(z_{t}*h_{t-1}\right). \end{array}\right. \end{array}$$

Due to the recurrent nature of LSTM and GRU layers, it is quite difficult for CPUs to accomplish their computation in parallel [27]. GPUs can explore little parallelism due to the branching operations [27]. Taking performance and energy efficiency into consideration, FPGA-based and ASIC-based accelerators can constitute a better choice.

Many studies demonstrated that fixed-point and dynamic fixed-point representations are an effective solution to reduce DNN model requirements for what concerns memory, computational units, power consumption and timing, without a significant impact on model accuracy [28–32]. FPGAs and ASICs are the only computing platforms that allow the customization of pipelined compute data paths and memory subsystems at the level of data type precision, taking maximum advantage of this kind of optimization techniques.

The process meant to change the representation of data from floating point to fixed point is called quantization, and it may be applied independently to

- Weights of the network
- Input data
- Output data

Additionally, approximation techniques can be applied to the non-linear activation functions within a Neural Network with the purpose of reducing hardware complexity for their execution [33]. As already stated, the intrinsic structure of RNNs requires the presence of closed loop paths, leading to additional constraints that make their quantization more complex with respect to other DNN models. Numerous studies already demonstrated that RNNs can take advantage of compression techniques as well as other kinds of models. In particular, different methods have been described to quantize weights and data during the training phase of the model [1, 13, 34–42] or through a re-training/fine-tuning process [31, 43, 44]. The results generally show the possibility to achieve comparable accuracy but with a reduced memory footprint and computational complexity, depending on the bit-width chosen for the fixed-point representation. The most effective memory footprint reduction is achieved by considering Binary, Ternary, or Quaternary Quantization [1, 34, 35, 45] where only 2–4 bits are used to represent weights and/or data. Quantization-aware training requires in-depth knowledge on model compression (model designers and hardware developers may not have such expertise), and it increases model design efforts and training time significantly [46]. Moreover, the original training code or the entire training data may not be shared with model compression engineers. For these reasons, a post-training quantization approach may be preferable in some real-world scenarios where the user wants to run a black-box floating-point model in low-precision [47]. Most of the works cited so far present their results only focusing the quantization effects on the model accuracy, while little attention is given on how the quantization strategies can meet architectural considerations when dealing with the design of hardware accelerators. On the other hand, different studies use a post-training quantization approach with the purpose to accelerate RNN inference on hardware platforms that go from CPUs [14, 24] to FPGAs [37, 48–50]. Typical strategy is to quantize the weights of the model only [48, 51] or to additionally quantize a part of the whole collection of intermediate signals [38]. This leads to the necessity to construct a floating-point-based hardware accelerator [27, 52], or an accelerator composed of both fixed-point and floating-point computational units [51]. To the best of our knowledge, few works in the literature give enough details on how to deal with the obstacles of RNNs post-training quantization when a full fixed-point-based hardware is implemented. The purpose of this work is exactly to present a new post-training quantization methodology, described in detail in order to give the designer useful guidelines toward the implementation of a fixed-point-based FPGA/ASIC hardware accelerator for RNN inference.

## 3. Methods

In this section, our quantization strategy is described in detail. The following methodology has been implemented as a software tool based on the Python Tensorflow 2 API [23]. The quantization tool takes as input an RNN floating-point model and gives as output the quantized version of that model, which can be accelerated on a hardware device exploiting fixed-point-arithmetic. More precisely, uniform-symmetric [32] quantization is used to convert each floating-point value *x* into its integer version *x*_int_, as shown in equation 3:

(3) $$\begin{array}{c} x_{\text{int}}=\text{round}\left(\frac{x}{{\text{LSB}}_{x}}\right). \end{array}$$

LSB_*x*_ is the value to be associated with the least significant bit for the two's complement (C2) representation of the integer *x*_int_, that will be processed by the hardware. The de-quantized floating-point value can then be obtained by multiplying *x*_int_ by LSB_*x*_. The LSB value for independent signals can be chosen as a power of two (depending on the precision desired for the representation) or determined by the number of bits wanted to represent those signals. Once the LSB values of the independent signals have been determined or chosen, the rules of fixed-point arithmetic must be considered in order to determine remaining LSB values:

(i) The sum operation can be applied on two integers having the same LSB value and the result will have that same LSB value
(ii) The product operation can be executed on numbers having different LSB values (LSB_*a*_, LSB_*b*_), but the result will have its LSB value determined by equation 4:
  (4) $$\begin{array}{c} {\text{LSB}}_{\text{prod}}={\text{LSB}}_{a}\cdot {\text{LSB}}_{b}. \end{array}$$

In the specific case of RNN quantization, additional constraints must be considered apart from the ones already stated. Indeed, the presence of closed loop paths requires some feedback signals (i.e., cell state *c*_*t*_ or cell output *h*_*t*_) to be modified before re-entering the LSTM/GRU cell. In general, we can consider the possibility to modify the LSB value of these signals through a specific multiplier applying equation 5:

(5) $$\begin{array}{c} {\text{LSB}}_{t-1}={\text{LSB}}_{t}\cdot M, \end{array}$$

where LSB_*t*−1_ and LSB_*t*_ are, respectively, the LSB values for the cell input and output signals; *M* is a multiplicative factor that lets LSB_*t*_ become coherent with previous timesteps execution. In the particular case of all LSB values being a power of two, and with the hypothesis of LSB values becoming smaller going from the input to the output of the cell, this loop operation can simply consist in a truncation applied on the fixed-point representation of the feedback signal (i.e., cutting out a certain amount of bits from the right side of the C2 string). By executing the truncation operation, the LSB value of a fixed-point number changes as shown in equation 6:

(6) $$\begin{array}{c} {\text{LSB}}_{\text{trunc}}=LSB_{x}\cdot 2^{b_{x}}, \end{array}$$

where LSB_*x*_ is the LSB value before truncation and *b*_*x*_ determines the number of bits to be truncated. Truncation is a very simple operation to be performed by a custom hardware accelerator designed for ASICs/FPGAs, bringing advantage in terms of resource utilization and power consumption with respect to the use of a generic multiplier. For this reason, from now on, we will keep the hypothesis that all the signals of the network will be characterized by power-of-two LSB values. Once the LSB_*x*_ value is known for all the signals within the network, the necessary bit-width for their fixed-point representation (*N*_bit_) can be calculated through equation 7:

(7) $$\begin{array}{c} \left\{\begin{array}{c} N_{\text{bit}}=\log_{2}\left(\frac{x_{\max}}{{\text{LSB}}_{x}}+1\right)+1\text{ if }x_{\max}\geq 0,\\ N_{\text{bit}}=\log_{2}\left(\frac{x_{\max}}{{\text{LSB}}_{x}}\right)+1\text{ if }x_{\max}<0, \end{array}\right. \end{array}$$

|*x*_max_| constitutes the maximum absolute value assumed by the generic signal *x* when running the model on the whole dataset or part of it. Thanks to the analysis of signals dynamics, the quantization tool is able to give information to the hardware designer on the necessary bit-width to exploit in each point of the network. This pre-analysis becomes particularly important when dealing with *c*_*t*_ and *h*_*t*_ signals within LSTM or GRU cells, since their dynamics are not known before the inference execution. On the other hand, at the output of activation functions, the signals dynamic is fixed. (*x*_max_ = 1) and the pre-analysis is not necessary. Further details are given in the next sections to clarify how our method works when applied specifically to an LSTM cell (Section 3.1) or a GRU cell (Section 3.2).

### 3.1. LSTM Quantization

Figure 3 shows the aliases given to the LSB values in each point of the LSTM cell.

Input vectors are quantized with LSB_in_ and multiplied by the matrices representing gates weights (quantized on LSB_weights_) through a scalar product operation performed by the Multiply and ACcumulate (MAC) block. The bias sum within each gate does not influence the LSB value, but biases must be a priori quantized with LSB_in_·LSB_weights_ respective to the fixed-point sum rule previously mentioned.

Successively, activation functions are applied, modifying the LSB value by a factor LSB_act_ (as it will become clear later). Finally, the cell state (quantized on LSB_state_) takes part in the calculations through the pointwise operations shown in the upper data-path. Activation functions have been approximated following a method similar to what is described in [33], where each function becomes a combination of linear segments. Each segment is characterized by two parameters:

- The inclination *a* (quantized with LSB_act_) that acts as a multiplicative factor on the activation function input
- A bias *ß* (quantized with LSB_in_·LSB_weights_ · LSB_act_) to be summed to the activation function output

In our case study, we chose to use 7 segments to approximate the sigmoid function (the same ones presented in [33]) and 9 segments to approximate the tanh function, like shown in Figure 4.

For a question of simplicity, we chose to use a unique LSB_act_ value for the *a* coefficients of both functions. The characterizing parameters chosen for the two approximated functions are summarized in Table 1 and obtained by fixing LSB_act_ = 2^−5^.

The various segments have been characterized so that the percentage error made by using our approximated functions rather than the original ones stays in the order of 1%.  Figure 5 shows the absolute error obtained on the output of the approximated functions compared with the output of the original functions, in the given input range [−6, 6].

It can be noticed that, once the thresholds of the activation functions have been defined, the dynamics of MAC output signals can be limited to reduce the necessary bit-widths for their representation (e.g., *x*_max_  = 5 before sigmoid).

Under the hypothesis that the LSB values at the output of the LSTM cell will be smaller than the input ones, truncation becomes essential to make the feedback loop consistent. In other words, thanks to the truncation operation, we can be sure that for subsequent timesteps of the RNN execution, input data (*x*_*t*_, *h*_*t*_) and cell state *c*_*t*_ will always be represented with a constant LSB value. This explains the presence of the State Truncation and Output Truncation blocks in Figure 3. Additional truncation blocks can be inserted in order to reduce intermediate signals bit-width, thus reducing the overall hardware occupancy and power consumption. We decided to add truncation blocks in the points highlighted in yellow in Figure 3, i.e., after *mul*_0_ pointwise multiplier and after the pointwise tanh operation. The orange dot located at the *mul*_1_ multiplier indicates a truncation operation that must be applied for the respect of the fixed-point sum computed at the successive pointwise adder. In other words, in correspondence with the orange dot, there is no degree of freedom for the designer, differently from what happens with the yellow dots.

Considering what has been discussed so far, the following equations must be verified for the correct LSTM computation on a fixed-point-arithmetic hardware:

(8) $$\begin{array}{c} \left\{\begin{array}{c} {\text{LSB}}_{\text{gate}}={\text{LSB}}_{\text{in}}\cdot {\text{LSB}}_{\text{weights}}\cdot {\text{LSB}}_{\text{act}},\\ {\text{LSB}}_{mul_{0}}={\text{LSB}}_{\text{state}}\cdot {\text{LSB}}_{\text{gate}}\cdot 2^{b_{mul}},\\ {\text{LSB}}_{mul_{1}}={\text{LSB}}_{mul_{0}}={\text{LSB}}_{{\text{state}}_{\text{out}}},\\ {\text{LSB}}_{\text{state}}={\text{LSB}}_{{\text{state}}_{\text{out}}}\cdot 2^{b_{\text{state}}},\\ {\text{LSB}}_{pw_{\tanh}}={\text{LSB}}_{{\text{state}}_{\text{out}}}\cdot {\text{LSB}}_{\text{act}}\cdot 2^{b_{\tanh}},\\ {\text{LSB}}_{mul_{2}}={\text{LSB}}_{pw_{\tanh}}\cdot {\text{LSB}}_{\text{gate}}. \end{array}\right. \end{array}$$

In summary, the parameters constituting our degrees of freedom are as follows:

- LSB_in_: The precision used to quantize LSTM inputs
- LSB_state_: The precision used to quantize the LSTM cellstate
- LSB_weights_: The precision used to quantize LSTM weights
- *b*_*mul*_, *b*_tanh_: The number of bits to truncate after *mul*_0_ multiplier and pointwise tanh, respectively

In Section 4, more details about the trade-off choices are given.

### 3.2. GRU Quantization

For what concerns the GRU cell, analogous considerations can be made for the starting conditions and for the approximation applied to the activation functions. Nevertheless, the sequence of operations is different and described with the new scheme shown in Figure 6.

In the GRU case, only one free truncation (yellow dot) can be individuated after the *mul*_1_ multiplier, while other three constrained truncation blocks (orange dots) are exploited.

The equations describing the quantized GRU cell behaviour are the following:

(9) $$\begin{array}{c} \left\{\begin{array}{c} {\text{LSB}}_{\text{gate}}={\text{LSB}}_{\text{in}}\cdot {\text{LSB}}_{\text{weights}}\cdot {\text{LSB}}_{\text{act}},\\ {\text{LSB}}_{mul_{0}}={\text{LSB}}_{\text{state}}\cdot {\text{LSB}}_{\text{gate}},\\ {\text{LSB}}_{mul_{1}}={\text{LSB}}_{\text{state}}\cdot {\text{LSB}}_{\text{gate}}\cdot 2^{b_{mul}},\\ {\text{LSB}}_{mul_{2}}={\text{LSB}}_{\text{gate}}^{2},\\ {\text{LSB}}_{\text{state}}={\text{LSB}}_{mul_{1}}\cdot 2^{b_{\text{state}}}. \end{array}\right. \end{array}$$

The parameters that constitute the degrees of freedom in this case are:

- LSB_in_: The precision used to quantize GRU inputs
- LSB_state_: The precision used to quantize the GRU state
- LSB_weights_: The precision used to quantize GRU weights
- *b*_*mul*_: The number of bits to truncate after *mul*_1_

In Section 4, more details about the trade-off choices are given.

## 4. Results

For the evaluation of our quantization method, we consider two models pretrained on the IMDb dataset for the sentiment classification task and two models pretrained on the Penn Treebank (PTB) dataset for the language modelling task. The results on the two datasets are treated separately in Section 4.1 and Section 4.2.

### 4.1. IMDb Results

The IMDb dataset contains 50000 different film reviews, and the task consists in distinguishing positive reviews from negative ones. The dataset was loaded from the Python Tensorflow library [23], limiting the vocabulary to the first 10000 most-used words. As an additional constraint, the length of each review was limited or padded to 235 words, which is the average review length in the given dataset.

The considered floating-point models are composed of

- An Embedding layer shrinking the input sequences from 235 elements to 32
- 32 LSTM or GRU cells
- A fully connected layer with one neuron producing the final binary output (positive/negative review)

The models were trained on a subset of 40000 reviews and tested on the remaining 10000, giving a test accuracy of 89.19% for the LSTM-based model and 90.24% for the GRU-based model. These values have then been compared to the accuracy obtained with two equivalently structured models where the LSTM/GRU layers have been quantized using the methodology described in Section 3.

#### 4.1.1. LSTM IMDb Results

The trade-off analysis has been carried out by acting on the following parameters: LSB_in_, LSB_state_, LSB_weights_, *b*_*mul*_, *b*_tanh_. For a matter of simplicity, only the most significant cases have been reported among all the possible combinations of these parameters. In particular, we considered cases characterized by:

- *b*_*mul*_ sized to have a precision equal to LSB_state_ at the output of the *mul*_0_ and *mul*_1_ pointwise multipliers. In this way, the operations are executed on the smallest number of bits allowed by the rules previously mentioned, and the State truncation block is unused
- *b*_tanh_ sized to preserve a precision equal to LSB_state_ at the output of the final pointwise tanh operation
- LSB_weights_ values ranging from 2^–10^ to 2^–2^ and LSB_in_, LSB_state_ values ranging from 2^−10^ to 2^−6^. These ranges were chosen by considering the accuracy trends obtained: bigger LSB values lead to accuracy values too low compared with the original one, while smaller LSBs do not cause additional benefit.

For a clearer understanding of the results, we compared the accuracy metric with the total reduction of the Memory Footprint (MF) needed for the hardware acceleration of the LSTM layer with the considered precision and truncation settings. The MF metric was determined considering two main contributions:

(i) Memory footprint needed for the weights of the network.
This can be estimated through equation 10:
  (10) $$\begin{array}{c} MF_{\text{weights}}=4\cdot \left(N_{\text{units}}+N_{\text{features}}\right)\cdot N_{\text{units}}+N_{\text{units}}, \end{array}$$
where *N*_features_ represents the number of elements composing the *x*_*t*_ input, and *N*_units_ indicates the number of cells used in the model (consisting in the dimension of the *h*_*t*_ vector as well).
(ii) Memory footprint needed for intermediate signals. In the hypothesis of building a hardware accelerator where a set of registers is located after each block shown in Figure 3 (i.e., cell inputs, gates output after truncation, pointwise operators result, cell state, cell output), this is the contribution of those registers on the total MF, considering the different bit-width *N*_bit_ of each signal.

As we noticed, the main contribution to the total MF is given by the weights. This means that the cases with the smallest MF are typically linked to bigger LSB_weights_ values.

Consequentially, we organized data by fixing the couples of values (LSB_state_, LSB_in_) and evaluating accuracy/MF values to varying of LSB_weights_.

The obtained curves are shown in Figure 7.

For a matter of clarity, some curves have been hidden from the figure since they had no particular trend compared to what is already shown, causing overlapping. We refer to the metrics of the floating-point model with the “FP” subscript (*MF*_*FP*_ and *Acc*_*FP*_), while the metrics concerning the quantized models are expressed with subscript “Q” (*MF*_*Q*_ and *Acc*_*Q*_).

Considering the various cases shown in the graph, we can see a MF reduction that goes from 64.1% to 89.4% compared with the floating-point model (*MF*_*FP*_ = 272 Kb), while the accuracy changes between the 0.3% and the 17% (*Acc*_*FP*_ = 89.19%).

We can also notice that the choice concerning weights precision (LSB_weights_) can, in most cases, lead to significant MF reductions at the cost of negligible accuracy loss. In particular, valuable results are met by setting LSB_weights_ = 2^−3^, leading to a 5-bits fixed-point representation for the weights of the layer.

The chosen settings for truncation become unfeasible when the LSB_state_, LSB_in_ values become bigger than 2^−7^. In these cases, a lighter truncation approach would be needed to achieve decent accuracy, but anyway obtaining results that are less efficient than most curves presented. The case giving the best accuracy/MF trade-off is characterized by (LSB_state_, LSB_in_, LSB_weights_) = (2^−10^, 2^−10^, 2^−3^), leading to *MF*_*Q*_ = 38.84 Kb (85.7% less than *MF*_*FP*_) and *Acc*_*Q*_ = 88.86% (0.33% less than *Acc*_*FP*_).

#### 4.1.2. GRU IMDb Results

In the case of the GRU-based model, the trade-off analysis has been carried out by acting on the following parameters: LSB_in_, LSB_state_, LSB_weights_, *b*_*mul*_.

The considered cases are characterized by

- *b*_*mul*_ sized to have a precision equal to LSB_gate_ at the output of the *mul*_1_ pointwise multiplier. This truncation setting was empirically justified by the evidence that the GRU model is more sensible to the precision given in its unique feedback path, thus requiring more bits
- LSB_weights_ values ranging from 2^–10^ to 2^–2^ and LSB_in_, LSB_state_ values ranging from 2^−10^ to 2^−6^ (same considerations made for the LSTM case study)

The MF metric was evaluated similarly to what was done with the LSTM, but with changes due to the different GRU cell scheme. In particular, the contribution of the weights is reduced (since only 3 gates are implemented), becoming:

(11) $$\begin{array}{c} MF_{\text{weights}}=3\cdot \left(N_{\text{units}}+N_{\text{features}}\right)\cdot N_{\text{units}}+N_{\text{units}}. \end{array}$$

The results are graphed in Figure 8 by varying LSB_weights_ with fixed couples of values (LSB_state_, LSB_in_).

Even for the GRU-based model, our quantization method leads to significant MF reduction (from 61.4% to 89.7%) with respect to the floating-point case (*MF*_*FP*_ = 204 Kb), while the accuracy changes between the 0.01% and the 14.3% (*Acc*_*FP*_ = 90.24%). The curves trends show a particular dependence from the LSB_state_ value, which must be smaller than 2^−8^ to find cases with an acceptable 1% accuracy drop. The best accuracy/MF trade-off is once again met by setting LSB_weights_ = 2^–3^. The best case is characterized by (LSB_state_, LSB_in_, LSB_weights_) = (2^–10^, 2^–10^, 2^–3^), giving *Acc*_*Q*_ = 90.23% (0.01% drop) and *MF*_*Q*_ = 34.94 Kb (82.9% reduction).

### 4.2. PTB Results

We extended our results on the Peen Tree Bank (PTB) corpus dataset [53], using the standard preprocessed splits with a 10 K size vocabulary. The dataset contains 929 K training tokens, 73 K validation tokens, and 82 K test tokens. The task consists in predicting the next word completing a sequence of 20 timesteps.

For fair comparison with existing works, we considered floating-point models composed of

- An Embedding layer shrinking the input features to 300
- 300 LSTM or GRU cells
- A Fully Connected layer with 10000 neurons producing the final label

The models were trained considering the Perplexity per word (PPW) metric, which is an index of how much “confused” the language model is when predicting the next word.

The PPW values obtained by testing the resulting models are 92.79 for the LSTM-based model and 91.33 for the GRU-based model. These values have then been compared to the perplexity obtained with two equivalently structured models where the LSTM/GRU layers have been quantized using the methodology described in Section 3.

#### 4.2.1. LSTM PTB Results

Keeping as a reference the discussion made in Section 4.1, the trade-off choices taken for the PTB LSTM-based model are listed below:

- *b*_*mul*_ sized to have a precision equal to LSB_state_ at the output of the *mul*_0_ and *mul*_1_ pointwise multipliers. In this way, the operations are executed on the smallest number of bits allowed by the rules previously mentioned, and the State truncation block is unused
- *b*_tanh_ sized to preserve a precision equal to LSB_state_ at the output of the final pointwise tanh operation
- LSB_weights_ values ranging from 2^–5^ to 2^5^ and LSB_in_, LSB_state_ values ranging from 2^–5^ to 2^0^. These ranges were chosen by considering the perplexity trends obtained: higher values deeply compromise the quality of the model. It can be noticed that they are different from the IMDb case study. This is explained by the different dynamics for input, state, and weights signals.

The obtained curves are shown in Figure 9.

From the graph, we can see a MF reduction that goes from 53.1% to 84.4% compared with the floating-point model (MF_FP_ = 22650 Kb), while the PPW changes between the 1% and the 38.5% (PPW_FP_ = 92.79). Even for the PTB case study, we can notice that the choice concerning weights precision (LSB_weights_) is the one that most of all determines MF reduction, at the cost of negligible increase in the PPW metric. On the other hand, LSB_in_ is the one affecting PPW metric the most: varying LSB_in_ while keeping LSB_state_ fixed actually generates widely spaced curves. The case we selected in simulation is characterized by (LSB_state_, LSB_in_, LSB_weights_) = (2^−5^, 2^−5^, 2^−1^), giving PPW_*Q*_ = 93.75 (0.96 greater than PPW_FP_) and *MF*_*Q*_ = 7789 Kb (65.6% reduction).

#### 4.2.2. GRU PTB Results

The chosen quantization/truncation settings are as follows:

- *b*_*mul*_ sized to have a precision equal to LSB_state_ at the output of the *mul*_1_ pointwise multiplier. Differently from what happened with the GRU model on IMDb, the PTB language modelling task allows us to use the minimum number of allowed bits without losing on the PPW metric
- *b*_tanh_ sized to preserve a precision equal to LSB_state_ at the output of the final pointwise tanh operation
- LSB_weights_ values ranging from 2^−5^ to 2^5^ and LSB_in_ values ranging from 2^−5^ to 2^3^, and LSB_state_ values ranging from 2^−5^ to 2^0^ (same considerations made for the LSTM PTB case study)

The obtained curves are shown in Figure 10.

In this case, the MF reduction goes from 59.4% to 87.5% compared with MF_FP_ = 16987.5 Kb, while the PPW changes between the 0.8% and the 9.2% (PPW_FP_ = 91.33). It must be noticed that some curves contain less points than others. This is due to the absence of cases where the combination of independent LSB values produces a LSB_gate_ value greater than 1, which cannot be used to properly represent signals whose dynamic is limited by sigmoid and tanh activation functions.

The simulation on the GRU-based model for the PTB task showed that it is possible to achieve PPW_*Q*_ values smaller (thus better) than PPW_FP_. This result implies that our post-training quantization can make the quality metric of a model improve with respect to its task. The best PPW/MF trade-off is met by setting (LSB_state_, LSB_in_, LSB_weights_) = (2^−1^, 2^2^, 2^0^), giving PPW_*Q*_ = 90.57 (0.76 less than PPW_FP_) and MF_*Q*_ = 4238.1 Kb (75.1% reduction).

## 5. Comparison with Related Works

In this section, we make a comparison between the results obtained with the proposed quantization method and the results from other works in the literature. To make the benchmark the most fair possible, we consider other manuscripts working with LSTM/GRU-based models used for the IMDb and PTB tasks.  Table 2, respectively, shows the similar results as Table 3 of the comparison. It must be considered that in this benchmark there may be no equivalence between models' structures or training strategies. For this reason, the focus of our comparison is not on the original floating-point accuracy/PPW, but rather on the variation of the metric when applying quantization.

In Table 2, we can notice that our method leads to smaller negative variations than most of other works shown, especially with regard to the GRU-based model. This advantage comes at the cost of larger bit-widths for weights or activations, mainly due to the different nature of the proposed methodology which is post-training rather than based on a quantization-aware training. Similar considerations can be made for the PTB case study in Table 3. The exception is our GRU-based model achieving better PPW than its floating-point version, which is a result obtained by few other works in this field.

Notice that the comparison is made in terms of bit-widths rather than MF reduction because other works do not actually consider the hardware application of the obtained quantized models. Our method, instead, is described considering the subsequent hardware implementation of our models on architectures completely based on fixed-point arithmetic.

## 6. Conclusions and Future Work

DNNs have become important tools for modelling non-linear functions in many applications. However, the inference of a DNN may lead to large storage size and runtime memory usage which impede their execution in on-the-edge applications, especially on resource-limited platforms or within area/power-constrained applications. To reduce plain feed forward DNN complexity, techniques such as quantization and pruning have been proposed during years. Nevertheless, little attention has been paid to relaxing the computational resource requirements of RNNs. This work proposes a detailed description of a new effective methodology for the Post-training quantization of RNNs. In particular, we focus on the quantization for LSTM and GRU RNNs, two of the most popular models for their performance in various tasks. Our quantization tool is compliant with the Python Tensorflow 2 framework and converts a floating-point pretrained LSTM/GRU model in its fixed-point version to be implemented on a custom hardware accelerator for FPGA/ASIC devices. The described methodology gives all the guidelines and rules to be followed in order to take maximum advantage of bit-wise optimizations within the accelerator design. We tested our quantization tool on models pretrained on the IMDb sentiment classification task and on the PTB language modelling task. The results show the possibility to obtain up to 90% memory footprint reduction with less than 1% loss in accuracy and even a slight improvement in the PPW metric when comparing each quantized model to its floating-point counterpart. We proposed a benchmark between our Post-training results and other works from the literature, noticing that they are mostly based on quantization-aware training. The comparison demonstrates that our algorithm affects models' accuracy in the same measure of other methods. This comes at the cost of bigger bit-widths for weights/activations representation but with all the advantages of a Post-training approach. In addition, our work is the only one taking into account the hardware implementation of a fully-fixed-point-based accelerator after quantization, which is a valuable approach to improve timing performance, resource occupation, and power consumption. Future work will focus on the hardware characterization of our techniques in order to quantify the architectural benefits with respect to floating-point accelerators. In addition, quantization results may be extended to other RNN algorithms or other tasks to further demonstrate the portability of our methods.

## Figures and Tables

**Figure 1:** Standard LSTM layer.

**Figure 2:** Standard GRU layer.

**Figure 3:** LSB values within the LSTM cell.

**Figure 4:** Approximated linear activation functions.

**Figure 5:** Absolute error given by using the approximated functions rather than of the original ones.

**Figure 6:** LSB values within the GRU cell.

**Figure 7:** LSTM quantization results on the IMDb dataset.

**Figure 8:** GRU quantization results on the IMDb dataset.

**Figure 9:** LSTM quantization results on the PTB dataset.

**Figure 10:** GRU quantization results on the PTB dataset.

**Table 1:** Approximated activation functions parameters.

Tanh		
Input interval	Output	
**x** ≥ 2.375	*y*=1	
1.5 ≤ **x** < 2.375	*y*=0.09375*x*+0.765625	
1 ≤ **x** < 1.5	*y*=0.28125*x*+0.484375	
0.5 ≤ **x** < 1	*y*=0.59375*x*+0.171875	
−0.5 ≤ **x** < 0.5	*y*=0.9375*x*	
−1 ≤ **x** < −0.5	*y*=0.59375*x* − 0.171875	
−1.5 ≤ **x** < −1	*y*=0.28125*x* − 0.484375	
−2.375 ≤ **x** < −1.5	*y*=0.09375*x* − 0.765625	
**x** < −2.375	*y*=−1	

Sigmoid		
Input interval		Output

**x** ≥ 5		*y*=1
2.375 ≤ **x** < 5		*y*=0.03125*x*+0.84375
1 ≤ **x** < 2.375		*y*=0.125*x*+0.625
−1 ≤ **x** < 1		*y*=0.25*x*+0.5
−2.375 ≤ **x** < −1		*y*=0.125*x*+0.375
−5 ≤ **x** < −2.375		*y*=0.03125*x*+0.15625
**x** < −5		*y*=0

**Table 2:** Comparison of quantization results on the IMDb dataset.

	Model	#Layers	#Units	Quantization method	Weights bits	Activation bits	FP model accuracy	Quantized model accuracy	Accuracy variation
[34]	LSTM	1	128	In-training	4	32	82.87	79.64	−3.23
[1]	LSTM	1	512	In-training	4	4	89.54	88.48	−1.06
[39]	LSTM	1	70	In-training	4	32	84.98	86.24	+1.26
[40]	LSTM	3	512	In-training	4	4	86.37	86.31	−0.06
Our work	LSTM	1	32	Post-training	5	14	**89.19**	**88.86**	−**0.33**
[34]	GRU	1	128	In-training	4	32	80.35	78.96	−1.39
[1]	GRU	1	512	In-training	4	4	90.54	88.25	−2.29
Our work	GRU	1	32	Post-training	5	20	**90.24**	**90.23**	−**0.01**

**Table 3:** Comparison of quantization results on the PTB dataset.

	Model	#Layers	#Units	Quantization method	Weights bits	Activation bits	FP model PPW	Quantized model PPW	PPW variation
[13]	LSTM	1	300	In-training	3	3	89.8	87.9	−1.9
[1]	LSTM	1	300	In-training	4	4	109	114	+5
[41]	LSTM	1	300	In-training	4	4	97	100	+3
[42]	LSTM	1	300	In-training	2	2	97.2	110.3	+13.1
Our work	LSTM	1	300	Post-training	11	10	**92.8**	**93.7**	**+0.9**
[13]	GRU	1	300	In-training	3	3	92.5	92.9	+0.4
[1]	GRU	1	300	In-training	4	4	100	102	+2
Our work	GRU	1	300	Post-training	8	3	**91.3**	**90.6**	−**0.7**

## Data Availability

The data used to support the findings of this study are included within the article.
